# Up-regulation of miR-34c-5p inhibits nasopharyngeal carcinoma cells by mediating NOTCH1

This article has been retracted.

**DOI:** 10.1042/BSR20200302

**Published:** 2020-06-15

**Authors:** Xin Xu, Haomin Yan, Le Zhang, Jing Liu, Yu Huang, Haoyu Cheng

**Affiliations:** 1 Department of Otolaryngology, Yan’an Hospital of Kunming City, Yunnan 650031, P.R. China; 2 Department of Hematology, Aerospace Center Hospital of Beijing, Beijing 100049, P.R. China

**Keywords:** MiR-34c-5p, nasopharyngeal carcinoma, NOTCH1

## Abstract

**Objective:** To explore the correlation between miR-34c-5p and NOTCH1 in nasopharyngeal carcinoma (NPC). **Materials and methods:** qPCR was employed to quantify miR-34c-5p and NOTCH1 mRNA in NPC, and Western blot to detect NOTCH1. MiR-34c-5p mimics/inhibitor and NOTCH1 siRNA were constructed to analyze the role of miR-34c-5p/NOTCH1 on the biological function of NPC cells. **Results:** NPC cells showed lower miR-34c-5p expression and higher NOTCH1 expression than normal cells, and up-regulating miR-34c-5p or inhibiting NOTCH1 could strongly suppress the epithelial–mesenchymal transition (EMT), proliferation, invasion and migration of NPC cells, and induce apoptosis in them. Up-regulating miR-34c-5p could inhibit NOTCH1, and miR-34c-5p was negatively correlated with NOTCH1. Rescue experiment results revealed that NOTCH1 up-regulation could counteract the changes of cell process induced by increased miR-34c-5p. **Conclusion:** MiR-34c-5p inhibits the growth of NPC by down-regulating NOTCH1, so up-regulating miR-34c-5p or down-regulating NOTCH1 may become the potential direction of NPC treatment.

## Introduction

Nasopharyngeal carcinoma (NPC) is an epithelial cancer type caused by nasopharyngeal mucosal lesions, which is classified into keratinizing squamous cell carcinoma, basaloid squamous cell carcinoma, and non-keratinizing squamous cell carcinoma according to histologic features [1]. NPC is one of the most common cancers in South China [2], and its inducements are relatively complicated. Birth history, family history of NPC, relatively short leukocyte telomere length, and Epstein–Barr virus (EBv) are risk factors for NPC [3–5]. Gene regulation is a crucial environment factor for the development and progression of NPC, so understanding the molecular mechanism in this process is beneficial for the development of NPC therapy.

MiR-34c is a 77-bp long non-coding RNA located on human chromosome 11, belonging to the miR-34 family, which can regulate cell process by binding to target gene sequence fragments. MiR-34c inhibits Bcl2 by pairing to the 3′ untranslated region (UTR) of Bcl2 gene, thus down-regulating the viability of laryngeal cancer cells and inducing apoptosis in them [6], and it enhances the cell sensitivity to cisplatin by suppressing the SOX9/β-catenin/c-Myc pathway. Moreover, miR-34c in low level is a risk factor for NPC patients [7]. MiR-34c is related with the development and progression of non-small cell lung carcinomas by regulating genes such as *AXL, Cdh1*, and *Fn1* [8,9], and it can also maintain endoplasmic reticulum homeostasis by down-regulating XBP1, thus regulating the tumor mechanism [10].

NOTCH1 and its dominant signaling pathway are important links in the development of many diseases. For instance, one study by Rice et al. [11] showed that knockout of NOTCH1 could suppress the tumorigenesis effect of prostate cancer cells in rats, and could also down-regulate the metastatic ability of prostate cancer and enhance the sensitivity of the cancer to drugs, and one study by Gan et al. [12], confirmed that NOTCH1 in high level would accelerate the malignant growth and epithelial–mesenchymal transition (EMT) of tongue cancer and suppress their apoptosis. Furthermore, one study by Li et al. [13] revealed that NOTCH1 prevented DNA damage and cell death through cascade reaction among ATM, CHK2 and p53, and one study by Fender et al. [14] revealed that NOTCH1 pathway promoted the EMT of colon cancer cells by regulating CD44, Slug, and Smad.

There are also previous studies confirming that increased NOTCH1 in NPC takes a part in the development of the NPC tumor [15], and miR-34c may be an inhibitor of NPC [16]. MiR-34c-5p is a mature spliceosome of miR-34c. In the present study, it was found through detection of NPC tissue samples that compared with corresponding non-tumor normal tissues, NPC tissues showed down-regulated miR-34c-5p and up-regulated NOTCH1, and it was also predicted through bioinformatics tools that NOTCH1 had sequence sites that can bind to miR-34c. At present, the relationship of miR-34c-5p/NOTCH1 axis in NPC and the regulatory mechanism of them remain unclear. Therefore, under such a situation, the present study would try to explore the correlation of miR-34c-5p/NOTCH1 axis with NPC by regulating the expression of the two factors in NPC.

## Materials and methods

### NPC patients

NPC tissue specimens were sampled from 74 patients diagnosed with NPC in the Yan’an Hospital Affiliated to Kunming Medical University, and 47 corresponding non-tumor normal tissue specimens were also sampled, and used as a control group. The inclusion criteria of the patients were as follows: patients diagnosed with NPC. Their exclusion criteria were as follows: patients with mental disease, patients with other comorbid tumors, patients who had received operation, chemotherapy, radiotherapy or antibiotic therapy, and patients unwilling to cooperate with the treatment. Tissue specimens were cut into sections, and stored in liquid nitrogen for later detection. The present study was conducted according to the principles of the Declaration of Helsinki. Written informed consents were obtained from all the participants, and the present study was also approved by the Ethics Committee of Yan’an Hospital Affiliated to Kunming Medical University.

### Cell transfection

Human nasal epithelial cells (HNECs) and NPC cells (SUNE1, CNE2, HK1, and HONE1) purchased from the American Type Culture Collection (ATCC) were cultured in 5% CO_2_ animal cell incubator at 37°C under a culture medium system containing Dulbecco’s modified Eagle’s medium (DMEM) (HyClone Company), 10% fetal bovine serum solution (Gibco Company), and 1% penicillin–streptomycin solution (100×, Solarbio Company). Subsequent experiments were carried out after the cells were cultured to reach 80–90% confluence.

Before transfection, the culture medium was replaced with a culture medium without fetal bovine serum, and on the day of transfection, the cells were seeded into a six-well plate at 1 × 10^5^ cells/well. The miR-34c-5p mimics, miR-34c-5p inhibitor, NC mimics, NC inhibitor, NOTCH1 siRNA, and NC siRNA vectors were all purchased from Shanghai Sangon Biotech Co., Ltd. The cell lines were transfected with a Lipofectamine 2000 transfection kit (Invitrogen, United States) in strict accordance with the kit instructions. After 8 h of transfection, the culture medium was replaced with fresh culture medium at 37°C/5%CO_2_.

### qPCR assay

Total RNA was extracted using the TRIzol method, and the optical density (OD) of the total RNA at 260–280 nm was detected using an ultraviolet spectrophotometer, and the RNA with OD_260_/OD_280_ > 1.8 was used for next experiment. Reverse transcription and PCR amplification and quantification were conducted with RNA using a FastKing one-step reverse transcription-fluorescence quantitative kit (Tiangen Biotech (Beijing) Co., Ltd., FP314) and ABI PRISM 7000 (Applied Biosystems, United States). The primers of miR-34c-5p and NOTCH1 mRNA were all designed and synthesized by Shanghai Sangon Biotech Co., Ltd. qPCR was carried out under a reaction system referring to the kit specification. The system consisted of 50 μl total volume containing 1.25 μl upstream primer, 1.25 μl downstream primer, 1.0 μl probe, 10 pg/μg RNA template, 5 μl of 50× ROX Reference Dye ROX, and RNase-free ddH_2_O added to adjust the volume. The reaction process included reverse transcription at 50°C for 30 min (one cycle) and pre-denaturation at 95°C for 3 min (one cycle), followed by 40 cycles of denaturation at 95°C for 15 s, and annealing at 60°C for 30 s. The results were analyzed using an ABI PRISM 7000 instrument, and the data were normalized using the 2^–ΔΔ*C*_t_^ method, with U6 and GAPDH as internal references.

### Western blot

Cell protein extract (1 ml) was adopted to lyse cells, and the cell solution was repeatedly pipetted until the cells were completely lysed. Then the cells were centrifuged at 1.6 × 10^4^ ***g*** for 15 min to take the supernatant, and the protein was separated through sodium dodecyl sulfate/polyacrylamide gel electrophoresis (SDS/PAGE), and transferred to a nitrocellulose (NC) membrane. The membrane was allowed to stand at room temperature for 1 h (blocked by 5% skim milk-phosphate buffer saline (PBS) solution). Subsequently, the protein to be detected was allowed to stand with β-actin antibody at 4°C overnight, and the NC membrane was washed with PBS solution three times, added with goat anti-rabbit secondary antibody (HRP conjugant), and then allowed to stand for 1 h at room temperature. Finally, the NC membrane was washed with PBS solution, and visualized by electrochemiluminescence (ECL) reagent. The internal reference protein was β-actin, and the relative expression level of the protein to be detected was recorded as the gray value of the band to be detected/the gray value of β-actin protein band.

NOTCH1, E-cadherin, N-cadherin, β-catenin, Vimentin, Caspase-3, Caspase-9, Bax, Bcl-2, β-actin primary antibodies and goat anti-rabbit secondary antibodies (HRP-conjugant) were all purchased from Shanghai Abcam Company.

### Transwell assay

Transfected cells were prepared into cell suspension through enzymolysis with trypsin, and seeded into the upper compartment containing 200 μl solution with 10% fetal bovine serum +1% DMEM at 2 × 10^4^ cells/well. The lower compartment was added with 500 μl DMEM containing 10% fetal bovine serum. After 2 h of cell culture, the fluid in the upper compartment was removed, and the cells on the chamber wall were wiped off. The cells on the other side of the Transwell chamber were immobilized for 20 min, and the Transwell chamber was stained with Crystal Violet for 15 min, and then rinsed with PBS solution. Photographs about cell migration were acquired under a 200-fold microscope. The cells in three randomly selected fields were counted, and the values were averaged, and taken as the number of cells penetrating the membrane. The experiment was repeated three times. Invasion was detected in the same way as above steps after 8% matrix gel was laid on the plate, and the number of cells per well was changed to 5 × 10^4^.

### MTT assay

Transfected cells were subjected to trypsin enzymolysis, and centrifuged to remove enzyme solution, and then added with a fresh culture medium, and pipetted to prepare cell suspension. The cells were seeded into four 96-well plates at 5 × 10^3^ cells/100 μl in each well, with three wells in each group. One plate was taken out every 24 h, added with 5 mg/ml MTT solution at 10 μl/well, and then cultured continuously for 1 h. Subsequently, the medium was removed, and the OD at 570 nm was measured using an enzyme mark instrument. The experiment was repeated three times, and a cell viability-time curve was drawn.

### Dual luciferase reporter gene assay

PmirGLO-NOTCH1-wt and pmirGLO-NOTCH1-mut vectors were constructed, and co-transfected into cells with miR-34c-5p mimics and NC mimics, respectively. After 48 h of transfection, the dual luciferase reporter gene (Promega) was used to determine the luciferase intensity in strict accordance with instructions.

### Statistical analysis

The above index data were input into SPSS20.0 (Asia Analytics Formerly SPSS China) and GraphPad Prism 6.0 for statistical analysis, and the experiment was repeated three times. Measurement data were expressed as the mean ± standard deviation (mean ± SD), compared between groups using the independent-samples *t* test, and compared among multiple groups using the one-way ANOVA. Post hoc pairwise comparison was carried out by the LSD *t* test, and Pearson correlation analysis was carried out to explore the correlation of miR-34c-5p and NOTCH1 mRNA. All data were analyzed using the two-tailed test, and 95% was used as the confidence interval. *P*<0.05 indicates a significant difference.

## Results

### Down-regulated miR-34c-5p and up-regulated NOTCH1 in NPC

In the present study, we collected 74 NPC tissue specimens and 47 corresponding non-tumor normal tissue specimens, and quantified miR-34c-5p and NOTCH1 mRNA in those specimens. Figure 1A,B showed that compared with corresponding non-tumor normal tissues, NPC tissues showed decreased miR-34c-5p level and increased NOTCH1 mRNA level. We also determined the levels of miR-34c-5p and NOTCH1 in HNECs and NPC cell lines (SUNE1, CNE2, HK1, and HONE1). Figure 1C,D showed that miR-34c-5p was lowly expressed in NPC cells, while NOTCH1 was highly expressed in them. Because miR-34c-5p showed the lowest expression and the second lowest expression in HK1 and CNE2 cells among those cells, respectively, HK1 and CNE2 cells were selected as research objects for the present study. We constructed miR-34c-5p mimics and miR-34c-5p inhibitor expression vectors, and transfected them into HK1 and CNE2 cells, and adopted the qPCR and Western blot to determine the level of NOTCH1 in the transfected cells. Figure 1E,F showed that up-regulation of miR-34c-5p could inhibit NOTCH1, while down-regulation of it could up-regulate NOTCH1. The above results revealed that miR-34c-5p was lowly expressed in NPC, while NOTCH1 was highly expressed in it, and miR-34c-5p may be involved in regulating NOTCH1.

**Figure 1:** Down-regulated miR-34c-5p and up-regulated NOTCH1 in NPC (**A**) MiR-34c-5p was down-regulated in NPC tissues. (**B**) NOTCH1 was up-regulated in NPC tissues. (**C**) MiR-34c-5p was down-regulated in NPC cells. (**D**) NOTCH1 mRNA was up-regulated in NPC cells. (**E**) NOTCH1 mRNA was negatively regulated by miR-34c-5p. (**F**) NOTCH1 protein was negatively regulated by miR-34c-5p. * indicates *P*<0.05; ** indicates *P*<0.01, and *** indicates *P*<0.001. Each assay was repeated three times.

### MiR-34c-5p promotes cell apoptosis and suppresses cell proliferation, migration, invasion, and EMT

In order to explore the effects of miR-34c-5p on NPC cells, we constructed miR-34c-5p mimics and miR-34c-5p inhibitor expression vectors to regulate miR-34c-5p in HK1 and CNE2 cells. The qPCR results (Figure 2A) revealed that the expression of miR-34c-5p was up-regulated in the miR-34c-5p mimics group, while the expression was down-regulated in the miR-34c-5p inhibitor group. We applied the Western blot assay to determine the expression of pro-apoptotic proteins (Caspase-3, Caspase-9, and Bax) and anti-apoptosis protein (Bcl2). Figure 2B showed that up-regulation of miR-34c-5p gave rise to an increase in the expression of Caspase-3, Caspase-9, and Bax, and a decrease in the Bcl2 expression, while its down-regulation gave rise to opposite effects. It was found that N-cadherin not only participated in cell invasion together with E-cadherin, but also regulated EMT together with Vinmentin, and β-catenin affected cell migration. The results of Western blot assay (Figure 2D) revealed that up-regulation of miR-34c-5p promoted E-cadherin, but inhibited N-cadherin, β-catenin, and Vimentin, and the results of Transwell assay (Figure 2C,F) also revealed that up-regulation of miR-34c-5p inhibited cell invasion and migration. Moreover, the results of MTT assay (Figure 2E) revealed that up-regulation of miR-34c-5p inhibited cell viability, while its down-regulation enhanced cell viability. The above results indicated that miR-34c-5p could promote cell apoptosis and inhibit cell proliferation, migration, invasion, and EMT.

**Figure 2:** MiR-34c-5p promotes cell apoptosis and suppresses cell proliferation, migration, invasion, and EMT (**A**) Expression of miR-34c-5p in each group. (**B**) Up-regulation of miR-34c-5p inhibited Bcl2, and promoted Caspase-3, Caspase-9, and Bax. (**C**) Up-regulation of miR-34c-5p suppressed cell migration. (**D**) Up-regulation of miR-34c-5p promoted E-cadherin, and inhibited N-cadherin, β-catenin, and Vimentin. (**E**) Up-regulation of miR-34c-5p suppressed cell viability. (**F**) Up-regulation of miR-34c-5p inhibited cell invasion. * indicates comparison with the NC group, *P*<0.05, and ** indicates comparison with the NC group, *P*<0.01. Each assay was repeated three times.

### NOTCH1 inhibits cell apoptosis and promotes cell proliferation, migration, invasion, and EMT

Because of the abnormal expression of NOTCH1 in NPC and the regulation of NOTCH1 by miR-34c-5p, NOTCH1 siRNA vectors were constructed in the present study to explore the role of NOTCH1 in NPC cells. The results are shown in Figure 3. The results showed that inhibition of NOTCH1 resulted in up-regulation of Caspase-3, Caspase-9, Bax, and E-cadherin and down-regulation of Bcl2, N-cadherin, β-catenin, and Vimentin, and inhibition of NOTCH1 resulted in a decrease in cell viability, migration, and invasion, which indicated that NOTCH1 inhibited cell apoptosis and promoted cell proliferation, migration, invasion, and EMT.

**Figure 3:** NOTCH1 inhibits cell apoptosis and promotes cell proliferation, migration, invasion, and EMT (**A**) Expression of NOTCH1 protein in each group. (**B**) Inhibition of NOTCH1 up-regulated Caspase-3, Caspase-9, and Bax, but down-regulated Bcl2. (**C**) Inhibition of NOTCH1 suppressed cell migration. (**D**) Inhibition of NOTCH1 up-regulated the expression of E-cadherin, and down-regulated the expression of N-cadherin, β-catenin, and Vimentin. (**E**) Inhibition of NOTCH1 suppressed cell viability. (**F**) Inhibition of NOTCH1 suppressed cell invasion. * indicates comparison with the NC siRNA group, *P*<0.05, and ** indicates comparison with the NC siRNA group, *P*<0.01. Each assay was repeated three times.

### MiR-34c-5p targets NOTCH1

It was found that there were sequence fragments on the 3′ UTR of NOTCH1 that bind to miR-34c-5p according to prediction through the TargetScan database. Co-transfection of NOTCH1-wt and miR-34c-5p mimics into NPC cells decreased the fluorescence activity of the cells, while other co-transfection combinations did not cause obvious change to the activity (Figure 4A,B). Pearson correlation analysis revealed that NOTCH1 mRNA was negatively correlated with miR-34c-5p (Figure 4C). The above results suggested that miR-34c-5p could targetedly inhibit NOTCH1 at the post-transcriptional level.

**Figure 4:** MiR-34c-5p inhibits NOTCH1 in a targeted manner (**A**) There were binding sites between NOTCH1 3′UTR and miR-34c-5p. (**B**) Co-transfection of NOTCH1-wt and miR-34c-5p mimics resulted in a decline in the fluorescence activity. (**C**) MiR-34c-5p was negatively related to NOTCH1 mRNA. ** indicates that in comparison with the NC mimics group, *P*<0.01. Each assay was repeated three times.

### Rescue experiment

The above results indicated that miR-34c-5p mimics could down-regulate NOTCH1, promote cell apoptosis, and inhibit cell proliferation, migration, invasion, and EMT. In order to verify that miR-34c-5p regulated cell biological processes through NOTCH1, we transfected miR-34c-5p mimics and NOTCH1+miR-34c-5p mimics into HK1 and CNE2 cells, respectively, to analyze and compare the cell changes. Figure 5 shows that compared with cells transfected with miR-34c-5p mimics, cells transfected with NOTCH1+miR-34c-5p mimics showed down-regulated Caspase-3, Caspase-9, Bax, and E-cadherin, but up-regulated Bcl2, N-cadherin, β-catenin, and Vimentin. Also, NOTCH1+miR-34c-5p mimics enhanced cell viability, migration, and invasion. The above results indicated that up-regulation of NOTCH1 could counteract apoptosis induced by miR-34c-5p mimics, and promote cell proliferation, migration, invasion, and EMT (Figure 6).

**Figure 5:** Rescue experiment (**A**) Compared with the miR-34c-5p mimics group, the NOTCH1+miR-34c-5p mimics group showed down-regulated Caspase-3, Caspase-9, and Bax, and up-regulated Bcl2. (**B**) Compared with the miR-34c-5p mimics group, NOTCH1+miR-34c-5p mimics group showed down-regulated E-cadherin, and up-regulated N-cadherin, β-catenin, and Vimentin. (**C**) Compared with the miR-34c-5p mimics group, the NOTCH1+miR-34c-5p mimics group showed enhanced cell viability. (**D**) Compared with the miR-34c-5p mimics group, the NOTCH1+miR-34c-5p mimics group showed intensified cell migration. (**E**) Compared with the miR-34c-5p mimics group, the NOTCH1+miR-34c-5p mimics group showed intensified cell migration. * indicates comparison with the miR-34c-5p mimics group, *P*<0.05, and ** indicates that in comparison with the miR-34c-5p mimics group, *P*<0.01. Each assay was repeated three times.

**Figure 6:** The mechanism of miR-34c-5p/NOTCH1 axis in regulating NPC MiR-34c-5p inhibited NOTCH1 mRNA by binding to NOTCH1 mRNA, and finally regulated the proliferation, invasion, migration, and EMT of NPC cells.

## Discussion

NPC is the cancer with the highest incidence among malignant otolaryngological tumors, which seriously compromises the daily life and health of patients. Studying the regulatory mechanism of NPC cells is helpful to the treatment of NPC. miRNA is one of the important members for regulation of NPC cells, and its regulation on downstream target genes is a crucial mechanism of regulating the NPC cells. In the present study, it was found through NPC tissue specimen detection that miR-34c-5p was down-regulated in the specimens, while NOTCH1 was up-regulated in them, so we speculated that the abnormal expression of miR-34c-5p and NOTCH1 may be related to the development of NPC. It was also found that inhibition of miR-34c-5p and overexpression of miR-34c-5p could give rise to up-regulation and down-regulation of NOTCH1, respectively. In addition, it was found that there were sequence fragments on 3′UTR of PTEN that bind to miR-34c-5p according to prediction through the TargetScan database. These results indicated that miR-34c-5p may participate in the regulation of NOTCH1 expression in NPC.

In order to analyze the relationship between miR-34c-5p and NOTCH1 and how this relationship affects the development of NPC, we constructed three vectors, miR-34c-5p mimics, miR-34c-5p inhibitor, and NOTCH1 siRNA, to change the expression of miR-34c-5p and NOTCH1 in NPC. When miR-34c-5p was up-regulated, NOTCH1 was down-regulated and the cell proliferation, migration, invasion, and EMT were weakened. Meantime, the cell apoptosis was intensified. In contrast, when miR-34c-5p was down-regulated, NOTCH1 was up-regulated and the cell proliferation, migration, invasion, and EMT were strengthened. Meantime, the cell apoptosis was weakened. In addition, down-regulation of NOTCH1 also led to an increase in cell apoptosis and a decrease in cell proliferation, migration, invasion, and EMT. Dual luciferase reporter gene assay confirmed that miR-34c-5p could bind to NOTCH1. The above results suggested that miR-34c-5p may inhibit the malignant growth and expansion of NPC cells by down-regulating NOTCH1. Rescue experiment results revealed that up-regulation of NOTCH1 could counteract apoptosis induced by miR-34c-5p mimics, and promote cell proliferation, migration, invasion, and EMT.

NOTCH1 protein is an essential part of tumor formation, and NOTCH pathway is a key pathway to regulate cell differentiation and self-renewal of stem cells [17]. NOTCH1 could inhibit downstream E-cadherin by activating Slug in mammary epithelial cells, and finally promote the epithelial cells transform to stromal cells [18], and it can down-regulate MEF2 by activating Snail1 in embryonal rhabdomyosarcoma, thus suppressing cell differentiation and intensifying the characteristics of stem cells in tumor cells [19]. In addition, the NOTCH1/Snail axis up-regulates the metastatic activity of non-small cell lung carcinoma by inhibiting E-adherin [20]. NOTCH1 also affects cell migration, invasion, and proliferation by regulating proteins such as β-catentin, NF-κB, p53, HIF-1α, MAPK, and cdc2 [21–25]. According to the results in this study, the effect of miR-34c-5p on NPC cells may be realized through a series of cascade reactions. In those cascade reactions, miR-34c-5p changes the activity of the functional protein downstream of NOTCH1 by regulating NOTCH1, and the change of the activity induces corresponding changes of cell biological function. Therefore, miR-34c-5p/NOTCH1 is an effective regulator of NPC cells.

The present study has discussed the role of miR-34c-5p/NOTCH1 axis in the pathogenesis of NPC, and it holds that miR-34c-5p can inhibit the malignant expansion of NPC cells caused by high expression of NOTCH1. Although the present study has described the mechanism of action of miR-34c-5p/NOTCH1 axis from the molecular level, the clinical value of miR-34c-5p and NOTCH1 still needs further evaluation. Considering the abnormal expression of miR-34c-5p and NOTCH1 in NPC, we will investigate whether the two can be applied to early diagnosis and prognosis evaluation of NPC in the future, and whether regulating miR-34c-5p/NOTCH1 axis is beneficial to the treatment of NPC. What is the reason, why miR-34c-5p is down regulated in NPC? Is there an upstream factor of miR-34c-5p that regulates miR-34c-5p expression in NPC?These questions are also worth discussing in future studies.

## Conclusion

The present study has studied the relationship between miR-34c-5p/NOTCH1 and NPC, and has found a possible mechanism of NPC. In this mechanism (Figure 6), miR-34c-5p inhibits cell proliferation, migration, invasion, and EMT and promotes cell apoptosis by targeting NOTCH1. Therefore, up-regulation of miR-34c-5p helps to alleviate the malignant growth and metastasis of NPC.

## Abbreviations

Bax: BCL2 Associated X, Apoptosis Regulator
Bcl2: BCL2 Apoptosis Regulator
DMEM: Dulbecco’s modified Eagle’s medium
EMT: epithelial–mesenchymal transition
GAPDH: Glyceraldehyde-3-Phosphate Dehydrogenase
HNEC: human nasal epithelial cell
HRP: horseradish peroxidase
LSD: Least Significant Difference
MTT: 3-(4,5-Dimethylthiazol-2-yl)-2,5-diphenyltetrazolium bromide
NOTCH1: Notch Receptor 1
NPC: nasopharyngeal carcinoma
OD: optical density
PBS: phosphate buffer saline
qPCR: Quantitative Real-time Polymerase Chain Reaction
SOX9: SRY-Box Transcription Factor 9
UTR: untranslated region
U6: U6 small nuclear RNA
XBP1: X-Box Binding Protein 1
